# Long noncoding RNA *UCA1* promotes cell growth, migration, and invasion by targeting miR‐143‐3p in oral squamous cell carcinoma

This article has been retracted.

**DOI:** 10.1002/cam4.2808

**Published:** 2020-03-04

**Authors:** Qingyun Duan, Mei Xu, Meng Wu, Xiong Zhang, Min Gan, Hongbing Jiang

**Affiliations:** ^1^ Jiangsu Key Laboratory of Oral Diseases Nanjing Medical University Nanjing Jiangsu China; ^2^ Department of Oral and Maxillofacial Surgery Affiliated Hangzhou First People's Hospital Medical College of Zhejiang University Hangzhou Zhejiang China; ^3^ Department of Ophtalmology Hangzhou Jianggan District People's Hospital Hangzhou Zhejiang China; ^4^ Department of Oral and Maxillofacial Surgery The Affiliated Huaian No.1 People's Hospital of Nanjing Medical University Huaian Jiangsu China; ^5^ Department of Oral and Maxillofacial Surgery The Affiliated Stomatological Hospital of Nanjing Medical University Nanjing Jiangsu China

**Keywords:** miR‐143‐3p, *MYO6*, oral squamous cell carcinoma, *UCA1*

## Abstract

**Background:**

The long noncoding RNA (lncRNA) urothelial carcinoma‐associated 1 (*UCA1*) is dysregulated in many types of tumors; however, its role in oral squamous cell carcinoma (OSCC) remains unclear. This study aims to determine the effect of lncRNA *UCA1* on OSCC.

**Methods:**

Fifty‐six paired OSCC and adjacent nontumorous tissues were collected and the levels of *UCA1*, miR‐143‐3p, and *MYO6* in the tissues were evaluated by qRT‐PCR. In in vitro experiments, cell viability, migration, and invasion were measured by, respectively, performing CCK‐8, wound healing, and transwell assays. The target relationships among *UCA1*, miR‐143‐3p, and *MYO6* were verified by dual‐luciferase assay. Western blot and immunohistochemistry were carried out to determine the protein levels. Xenograft mouse model was established to explore the effects of *UCA1* in vivo.

**Results:**

Levels of *UCA1* and *MYO6* were increased significantly in OSCC, while the level of miR‐143‐3p was decreased compared with the adjacent nontumorous tissues. *UCA1* promoted OSCC cell growth, migration, and invasion both in vitro and in vivo, while miR‐143‐3p reversed the progression. *MYO6* was validated as a target for miR‐143‐3p, and *MYO6* overexpression reversed the effects of miR‐143‐3p mimic on OSCC cells.

**Conclusion:**

LncRNA *UCA1* contributes to the proliferation and metastasis of OSCC cells by targeting miR‐143‐3p and upregulating its downstream gene *MYO6*. *UCA1* could serve as a promising novel target therapy for treatment of OSCC.

## Graphical abstract

Our study indicates that the *UCA1* expression was significantly elevated in OSCC tissues and cells and was correlated with the metastasis and recurrence of OSCC patients. Moreover, the overexpression of *UCA1* markedly promoted OSCC progression in vitro and in vivo by upregulating *MYO6* expression as a sponge of miR‐143‐3p.

## 1 INTRODUCTION

Oral squamous cell carcinoma (OSCC) is the sixth most prevalent malignancy in the world,^1^ and often occurs in the lips, tongue, buccal mucosa, floor, gingiva, hard palate, and retromolar trigone.^2^ A study indicates that young white population aged 18‐44 years have a higher rate of developing OSCC.^3^ Though efforts have been made in advancing the diagnosis and treatment methods, 5‐year survival rate of patients with OSCC is still not satisfactory.^4^ Therefore, OSCC treatments, including extending survival time, remain a challenge to be solved.

Long noncoding RNAs (lncRNAs) can form complex networks by the interactions with microRNAs (miRNAs), messenger RNAs (mRNAs), and proteins, and play pivotal roles in different cancers.^5^ LncRNAs are involved in the progress of OSCC through affecting various aspects of cellular homeostasis.^6^ LncRNA urothelial cancer‐associated 1 (*UCA1*) exerts critical effects on various cancers. LncRNA *UCA1* is elevated in the bile duct carcinoma (BDC) and promotes BDC cell migration and invasiveness.^7^ Moreover, lncRNA *UCA1* can promote human pancreatic ductal adenocarcinoma stem cell properties and suppress tumor growth.^8^ The oncogenic role of lncRNA *UCA1* in other cancers, including glioblastoma,^9^ bladder,^10^ gastric,^11^ and prostate cancer,^12^ has been reported, the function of *UCA1* in OSCC remains to be elucidated.

MiRNAs can also function vitally in the posttranscriptional regulation through binding to the 3’UTR of mRNAs. It is revealed that miRNAs can be separated by lncRNAs from their target mRNAs.^13^ MiR‐143‐3p shows a tumor‐suppressive role in many cancers such as cervical cancer,^14^ osteosarcoma,^15^ colorectal cancer,^16^ and laryngeal squamous cell carcinoma 17; however, whether miR‐143‐3p has a tumor‐suppressive function in OSCC remains unclear.

Myosin VI (*MYO6*), which is widely expressed in various organisms and tissues, is a unique member of the myosin superfamily.^18^ *MYO6* could serve as an oncogene in human cancers, for instance, knocking down *MYO6* suppresses the growth and induces the apoptosis in prostate cancer, colorectal cancer, and gastric cancer.^19^, ^20^, ^21^ In addition, knockdown of *MYO6* also inhibits the proliferation of OSCC cells.^22^ Although *MYO6* has been reported in many human tumors, including OSCC cells, its role in OSCC is unknown.

In the current study, we explore the clinical characteristics and role of lncRNA *UCA1* in OSCC. We demonstrated that *UCA1* was markedly increased in OSCC tissues and cells, and that *UCA1* facilitated the progression of OSCC via regulating the miR‐143‐3p/MYO6 axis.

## 2 MATERIALS AND METHODS

### 2.1 Clinical tissues and cell lines

The tissues and matched adjacent normal tissues were collected from 56 OSCC patients (males/females, aged between 32 and 24 years, with a median age of 46 years) at the Affiliated Hangzhou First People's Hospital, Medical College of Zhejiang University from December 2016 to December 2017. The written informed consent was signed by all patients. The experiments were conducted following the ethical standards and were approved by the Affiliated Hangzhou First People's Hospital, Medical College of Zhejiang University, approval number: AHFPH20161221.

Human normal oral cell line HGF‐1 and OSCC cell lines (YD‐38, MK‐1) were obtained from the American Type Culture Collection (ATCC) and Cell Bank (Shanghai, China). The cells were grown in RPMI‐1640 medium containing 10% heat‐inactivated fetal bovine serum (Gibco) and 1% penicillin‐streptomycin (Gibco) at 37°C with 5% CO_2_.

### 2.2 Cell transfection

For cell transfection, YD‐38 cells (3 × 10^4^/mL) were transfected with negative control (NC) small interfering (si) RNAs, *UCA1* siRNA (si‐UCA1, Ribobio), *MYO6* siRNA (si‐MYO6, Ribobio), or co‐transfected with si‐UCA1/si‐MYO6 and miR‐143‐3p inhibitor, or miR‐NC inhibitor (GenePharma). MK‐1 cells (3 × 10^4^/mL) were transfected with a blank pcDNA3.1 vector (Invitrogen), a pcDNA3.1 containing *UCA1* expression plasmid (pc‐UCA1) or *MYO6* plasmid (*MYO6*), or co‐transfected with pc‐UCA1/MYO6 and miR‐143‐3p mimics, or miR‐NC mimics (GenePharma) using Lipofectamine 2000 (Invitrogen). The final concentration of vectors and miRNAs was 100 nmol/L. After transfection for 48 hours, the cells were preserved for the subsequent assays.

### 2.3 Reverse transcription‐quantitative polymerase chain reaction (RT‐qPCR)

Total RNA was extracted from OSCC tissues and cells by RNAiso Plus (Takara). To determine the levels of lncRNA, miRNA, and mRNA, the cDNA was obtained by RNA using RevertAid First Strand cDNA Synthesis Kit (Thermo Fisher Scientific). The reaction was performed on ABI PRISM 7900HT system (Applied Biosystems) with SYBR Premix Ex Taq (Takara). The levels of *UCA1*/mRNA and miR‐143‐3p were normalized to *GAPDH* and *U6*, respectively. The primers used are listed in Table 1 and the relative expressions were calculated by the 2^−ΔΔCt^ method.^23^

**Table 1:** Primers and sequences of qRT‐PCR

Gene	sequence (5′‐3′)
*UCA1*‐Forward	TGACAACAGATAACCACCT
*UCA1*‐Reverse	TCCGTATAGAAGACCACCTA
miR‐143‐3p‐Forward	GGGGTGAGATGAAGCACTG
miR‐143‐3p‐Reverse	CAGTGCGTGTCGTGGAGT
*MYO6*‐Forward	CAGAGCAACGTGCTCCAAAGTC
*MYO6*‐Reverse	GAAGCGTTGCTG TCGGTTCA
MMP‐2‐Forward	TGATTCTGGTCGCTCAGATG
MMP‐2‐Reverse	CTTGTTTCCCAGGAAGGTGA
MMP‐9‐Forward	AGGACCATGGGGATCCTTAC
MMP‐9‐Reverse	AACACAAGGCTGCCCATTAC
E‐cadherin‐Forward	TAACCGATCAGAATGAC
E‐cadherin‐Reverse	TTTGTCAGGGAGCTCAGGAT
N‐cadherin‐Forward	CAACTTGCCAGAAAACTCCAGG
N‐cadherin‐Reverse	ATGAAACCGGGCTATCTGCTC
U6‐Forward	CTCGCTTCGGCAGCACATA
U6‐Reverse	AACGATTCACGAATTTGCGT
GAPDH‐Forward	CACCATTGGCAATGAGCGGTTC
GAPDH‐Reverse	AGGTCTTTGCGGATGTCCACGT

### 2.4 Differential gene expression analyses

The http://www.ncbi.nlm.nih.gov/geo/query/acc.cgi?acc=GSE54672 dataset including one primary tumor tissue and one metastasis tissue was downloaded from the GEO. The differentially expressed genes (DEGs) were identified by interactive online tool GEO2R, with *P* < .05 and log fold‐change (FC) >2 served as the cutoff criteria. Venny 2.1 was used to identify the overlapping DEGs, which were upregulated in the http://www.ncbi.nlm.nih.gov/geo/query/acc.cgi?acc=GSE54672, TargetScan7.2 datasets, and miRanda datasets.

### 2.5 Dual‐luciferase reporter assay

The binding site between *UCA1* and miR‐143‐3p was determined by starbase v3.0 and that between *MYO6* and miR‐143‐3p was predicted by TargetScan7.2. The *UCA1* and *MYO6* wt/mut 3′‐UTR were, respectively, inserted into pmirGLO plasmid (Promega). Then, the vectors (2 µg/mL) were co‐transfected with miR‐NC or miR‐143‐3p mimics (50 nmol/L) into the cells using Lipofectamine 2000 reagent (Invitrogen). Luciferase activity was measured by the Dual‐Glo Luciferase assay (Promega).

### 2.6 Cell counting kit‐8 (CCK‐8) assay

Cell growth was detected using CCK‐8 (Dojindo). Briefly, YD‐38 and MK‐1 cells (5 × 10^3^/well) were incubated for 24 or 48 hours. Then, CCK‐8 solution was added and incubated for another 4 hours. The optical density (OD) was measured at 490 nm using a microplate reader (Detie Laboratory Equipment Companya).

### 2.7 Wound healing assays and Transwell invasion assay

The transfected cells (1 × 10^5^/well) were cultured in 6‐well plates until the cell confluence reached over 90%, and then a scratch was created using a 10‐μL pipette tip. The wound closures were observed and photographed at 0 and 24 hours after scratching under a microscope (Olympus). The wound closure was measured by ImageJ (v1.42, NIH).

To detect the invasive ability of OSCC cells, transwell chamber was treated with Matrigel (BD Biosciences). Next, the transfected cells (1 × 10^5^ cells/well) were seeded into the upper chamber containing serum‐free medium, while 600‐μL medium was added into the lower chamber. After incubation for 24 hours, the invaded cells were fixed, stained, and counted under a microscope (Olympus).

### 2.8 Western blot

The protein in tissues and cells was isolated in RIPA lysis buffer (Beyotime) and the concentration of protein was measured using BCA Kit (Beyotime). An equal amount of proteins were separated on 10% SDS‐PAGE (40 µg protein/lane) and then were transferred onto PVDF membranes (Millipore), which were incubated in 5% nonfat milk for 1 hour at room temperature. The membranes were subsequently incubated at 4°C overnight with primary antibodies including anti‐MYO6 (1:1000, ab230478, Abcam), anti‐MMP‐2 (1:1000, ab37150, Abcam), anti‐MMP‐9 (1:1000, ab38898, Abcam), anti‐GAPDH (1:1000, ab8245, Abcam), anti‐E‐cadherin (1:1000, #3195, Cell Signaling Technology), and anti‐N‐cadherin (1:1000, #13116, Cell Signaling Technology). Next, they were incubated with the HRP‐conjugated goat anti‐rabbit IgG (1:10 000, ab6721, Abcam) for 1 hour at room temperature. The bands were detected by enhanced chemiluminescence detection kit (Thermo scientific), and the intensity was quantified using ImageJ software v1.42 (NIH). The GAPDH served as a loading control.

### 2.9 Immunohistochemistry

After immersing the sections in citrate (pH = 6.0) and antigen retrieval buffers, the paraffin‐embedded sections were treated with 3% H_2_O_2_ and incubated with 10% goat serum. After that, the sections were washed with Tris‐buffered saline Tween‐20 (TBST) and then incubated with rabbit polyclonal anti‐MYO6 (1:100, ab230478, Abcam) at 4°C overnight. Next, the sections were incubated with HRP‐conjugated goat anti‐rabbit IgG. The signal was detected by DAB Substrate kit following the manufacture's instruction and the images were observed under a microscope (Olympus).

### 2.10 Xenograft animal model

Male nude mice (aged 4‐6 weeks old; weighting 20‐24 g) were purchased from Slac Laboratory Animal Center (Shanghai, China) and housed in an SPF‐grade barrier environment at the Affiliated Hangzhou First People's Hospital, Medical College of Zhejiang University, approval number: AHFPH20171230. The animal protocol was approved by the Institutional Animal Care and Use Committee of the Affiliated Hangzhou First People's Hospital, Medical College of Zhejiang University. The transfected cells (5 × 10^7^/mL, 0.1 mL) were subcutaneously injected into the nude mice (n = 5 per group). Four weeks later, the mice were sacrificed and the tumor tissues were photographed, weighed, and collected for immunohistochemistry and Western blot.

### 2.11 Statistical analysis

GraphPad Prism version 5.0 (GraphPad Software) was used to analyze the data, which were shown as the mean ± standard deviation (SD). Student's *t* tests were used to examine differences between the two groups, whereas differences between three or more groups were analyzed by one‐way ANOVA. The significance of correlations among *UCA1*, miR‐143‐3p, and *MYO6* levels was assessed by the Pearson correlation coefficient. A *P* < .05 was considered as statistically significant. All experiments were repeated at least in triplicate.

## 3 RESULTS

### 3.1 *UCA1* is upregulated in OSCC and sponges miR‐143‐3p

To explore whether *UCA1* is abnormal in OSCC, we measured the level of *UCA1* in 56 OSCC tissues and matched normal ones. The level of *UCA1* was increased more in the tumor tissues than that in normal tissues (*P* < .001, Figure 1A); however, the level of miR‐143‐3p exhibited an opposite trend (*P* < .001, Figure 1B), showing a notably negative correlation with *UCA1* expression (*P* < .001, Figure 1C). Similarly, the *UCA1* showed a higher level in the two OSCC cell lines than that in human normal oral cells, while miR‐143‐3p had an opposite expression (*P* < .01, Figure 1D,E).

**Figure 1:** The level of lncRNA *UCA1* is increased and that of miR‐143‐3p is reduced in OSCC, and lncRNA *UCA1* is a sponge of miR‐143‐3p. The levels of lncRNA *UCA1* (A) and miR‐143‐3p (B) were determined in OSCC tissues and adjacent noncancerous tissues by qRT‐PCR. C, Scatter diagram revealed a negative correlation between *UCA1* and miR‐143‐3p in 56 pairs of OSCC tissues by RT‐qPCR. The lncRNA *UCA1* (D) and miR‐143‐3p (E) were detected in OSCC cell lines and human normal oral cell line by RT‐qPCR.(F) The miR‐122 binding position on *UCA1* was predicted by starbase v3.0. G and H, Dual‐luciferase reporter assay of OSCC cells co‐transfected with wt/mut *UCA1* sequence and miR‐143‐3p mimics or the miR‐NC. ^**^ *P* < .01

To further assess the clinical significance of *UCA1* expression in OSCC, the OSCC patients were assigned into high (n = 25) and low (n = 31) expression groups according to the median level of expression. As shown in Table 2, high *UCA1* expression was remarkably correlated with lymphatic metastasis and recurrence. We also evaluated the clinical significance of miR‐143‐3p in OSCC. We found that low level of miR‐143‐3p was significantly related to lymphatic metastasis and recurrence (Table 3).

**Table 2:** The relationship between *UCA1* expression and clinical characteristics of oral squamous cell carcinoma

Characteristics	Patients (n = 56)	*UCA1*		*χ^2^*	*P*
		High (n = 25)	Low (n = 31)		
Age					
≤60	30	13 (43.33%)	17 (56.67%)	0.045	.832
>60	26	12 (46.15%)	14 (53.85%)		
Sex					
Male	32	14 (43.75%)	18 (56.25%)	0.024	.877
Female	24	11 (45.83%)	13 (54.17%)		
Lymphatic metastasis					
Present	23	14 (60.87%)	9 (39.13%)	4.159	.041
Absent	33	11 (33.33%)	22 (66.67%)		
Recurrence					
Present	18	12 (66.67%)	6 (33.33%)	5.206	.023
Absent	38	13 (34.21%)	25 (65.79%)		
Absent	38	24 (63.16%)	14 (36.84%)		

**Table 3:** The relationship between miR‐143‐3p expression and clinical characteristics of oral squamous cell carcinoma

Characteristics	Patients (n = 56)	miR‐143‐3p		*χ^2^*	*P*
		High (n = 30)	Low (n = 26)		
Age					
≤60	30	15 (50.00%)	15 (50.00%)	0.331	.565
>60	26	15 (57.69%)	11 (42.31%)		
Sex					
Male	32	17 (53.13%)	15 (46.87%)	0.006	.938
Female	24	13 (54.17%)	11 (45.83%)		
Lymphatic metastasis					
Present	23	8 (34.78%)	15 (65.22%)	5.540	.019
Absent	33	22 (66.67%)	11 (33.33%)		
Recurrence					
Present	18	6 (33.33%)	12 (66.67%)	4.368	.037
Absent	38	24 (63.16%)	14 (36.84%)		

*UCA1* has been reported as ceRNAs to specific miRNAs in regulating tumor progression. Here, starbase v3.0 identified that *UCA1* had a complementary binding site with miR‐143‐3p (Figure 1F). Furthermore, the miR‐143‐3p mimics obviously suppressed the luciferase activity of the vector containing *UCA1*‐WT (*P* < .01); however, it had no effect on that of the vector with *UCA1*‐Mut in YD‐38 and MK‐1 cells (Figure 1G,H).

### 3.2 MiR‐143‐3p reverses the *UCA1*‐induced OSCC cell proliferation, migration, and invasion

To validate our speculation that *UCA1* promotes proliferation, migration, and invasion of OSCC cells by acting as a sponge of miR‐143‐3p, the *UCA1* and miR‐143‐3p expressions in transfected cells were determined. The *UCA1* expression was notably decreased by si‐UCA1 but were increased in the cells transfected with pc‐UCA1 (*P* < .01); meanwhile, the miR‐143‐3p mimics or inhibitors had no significant effects on the *UCA1* expression (Figure 2A,B). In addition, the levels of miR‐143‐3p in si‐UCA1 group and mimic group were upregulated but could be inhibited by pc‐UCA1 and inhibitors (*P* < .01, Figure 2C,D). The CCK8 assay results showed that compared with the controls, knocking down *UCA1* in YD‐38 cells significantly suppressed the cell viability, which, however, was rescued by the miR‐143‐3p inhibitors (*P* < .05, Figure 2E). In MK‐1 cells, the overexpressed *UCA1* greatly promoted cell proliferation, and miR‐143‐3p mimics attenuated the effect of *UCA1* (*P* < .05, Figure 2F).

**Figure 2:** LncRNA *UCA1* promotes OSCC cell proliferation, migration, and invasion by inhibiting miR‐143‐3p. A and B, The lncRNA *UCA1* expression in YD‐38 and MK‐1 cells 48 h after transfection was determined by RT‐qPCR. C and D, The miR‐143‐3p expressions in YD‐38 and MK‐1 cells 48 h after the transfection were determined by RT‐qPCR. E and F, CCK‐8 assays of YD‐38 and MK‐1 cell proliferation at 24 h and 48 h. G and H, Representative images of cell migration in each group of YD‐38 and MK‐1 cells at 0 h and 24 h. I and J, Representative images of cell invasion in each group of YD‐38 and MK‐1 cells at 24 h. K and L, Migration distance in each group of YD‐38 and MK‐1 cells. M and N, The number of invasive cells in each group of YD‐38 and MK‐1 cells. ^*^ *P* < .05, ^**^ *P* < .01

To further investigate the effect of *UCA1* on metastasis, wound healing and transwell assays were performed (Figure 2G‐J). The inhibition of *UCA1* by siRNA effectively suppressed cell migration and invasion, while overexpressed *UCA1* greatly accelerated the migration and invasion in comparison to those in control groups; however, these effects of *UCA1* were reversed by miR‐143‐3p (*P* < .01, Figure 2K‐N).

### 3.3 *UCA1* positively regulates *MYO6* by sponging miR‐143‐3p

The genes that were potentially regulated by miR‐143‐3p were determined. For the http://www.ncbi.nlm.nih.gov/geo/query/acc.cgi?acc=GSE54672 dataset, a total of 2232 upregulated DEGs were extracted, and 17 DEGs, including *MYO6*, had overlapping area in the three databases (Figure 3A). The targeted binding site between miR‐143‐3p and *MYO6* was predicted by TargetScan7.2 (Figure 3B), and luciferase reporter assays verified that miR‐143‐3p mimics markedly reduced the luciferase activity in the *MYO6*‐wt group but it had no effect on the *MYO6*‐mut group in YD‐38 and MK‐1 cells (Figure 3C,D). The protein and mRNA levels of *MYO6* were detected by Western blot and RT‐qPCR in transfected OSCC cells. The pc‐UCA1 or miR‐143‐3p inhibitors increased *MYO6*, which was significantly suppressed by si‐UCA1 or miR‐143‐3p mimics (*P* < .01, Figure 4A‐F). The *MYO6* expression in co‐transfected cells exhibited no significant difference from that in the control group. Moreover, the RT‐qPCR and immunohistochemistry results showed that *MYO6* in the OSCC tissues was greatly elevated compared with that in normal tissues (*P* < .01, Figure 4G‐I). We found that *MYO6* was negatively correlated with miR‐143‐3p but positively correlated with *UCA1* in 56 pairs of OSCC tissues by qRT‐PCR (*P* < .001, Figure 4J,K).

**Figure 3:** MiR‐143‐3p directly targets *MYO6* in OSCC cells. A, The http://www.ncbi.nlm.nih.gov/geo/query/acc.cgi?acc=GSE54672 dataset, miRDB website, and Targetscan website were used to predict the overlapped mRNA of miR‐143‐3p. B, The predicted miR‐143‐3p binding site in the *MYO6* using Targetscan7.2. C and D, Dual‐luciferase reporter assay of OSCC cells co‐transfected with wt/mut *MYO6* and miR‐143‐3p mimics or the miR‐NC. ^**^ *P* < .01

**Figure 4:** *MYO6* is elevated in OSCC. A, Western blot of *MYO6* in each group of YD‐38 cells. B, The protein levels of the *MYO6* in YD‐38 cells. C, The mRNA expression of *MYO6* in each group of YD‐38 cells. D, Western blot of *MYO6* in each group of MK‐1 cells. E, The protein levels of the *MYO6* in MK‐1 cells. F, The mRNA expression of *MYO6* in each group of MK‐1 cells. G, The *MYO6* was detected in OSCC tissues and adjacent noncancerous tissues by qRT‐PCR. H, Representative immunohistochemical images of OSCC tumor sections for *MYO6* (scale bar = 100 μm). I, The staining intensity of *MYO6* by immunohistochemistry. J and K, Scatter diagram showed a positive correlation of *UCA1* and *MYO6* and a negative correlation of miR‐143‐3p and *MYO6* in 56 pairs of OSCC tissues by RT‐qPCR. ^*^ *P* < .05, ^**^ *P* < .01

### 3.4 *MYO6* promotes OSCC cell proliferation and metastasis in vitro

To confirm the effect of *MYO6* on the OSCC progression, *MYO6* expression in OSCC cells was determined at the protein and mRNA levels. The knockdown of *MYO6* in YD‐38 cells and overexpression of *MYO6* in MK‐1 cells were effective, and miR‐143‐3p reversed the expression tendency of *MYO6* (*P* < .01, Figure 5A‐F).

**Figure 5:** MiR‐143‐3p negatively regulates *MYO6* in OSCC cell lines. A, Western blot analysis of *MYO6* in each group of YD‐38 cells. B, The protein expression of the *MYO6* in YD‐38 cells. C, The mRNA expression of *MYO6* in each group of YD‐38 cells. D, Western blot analysis of *MYO6* in each group of MK‐1 cells. E, The protein expression of the *MYO6* in MK‐1 cells. F, The mRNA expression of *MYO6* in each group of MK‐1 cells. ^*^ *P* < .05, ^**^ *P* < .01

The CCK‐8 results showed that proliferation of YD‐38 cells was sharply inhibited by the knockdown of *MYO6* but significantly increased by miR‐143‐3p inhibitors (*P* < .01, Figure 6A). Moreover, the MK‐1 cell growth was greatly improved by overexpressing *MYO6* but suppressed by miR‐143‐3p mimics (*P* < .01, Figure 6B). Similarly, the inhibitory effect of miR‐143‐3p on cell migration and invasion was also rescued by *MYO6* (*P* < .01, Figure 6C‐J).

**Figure 6:** MiR‐143‐3p inhibits OSCC cell proliferation, migration, and invasion by inhibiting *MYO6*. A and B, CCK‐8 assays of YD‐38 and MK‐1 cell proliferation in each group at 24 and 48 h. C and D, Representative images of cell migration in each group of YD‐38 and MK‐1 cells at 0 and 24 h. E and F, Representative images of cell invasion in each group of YD‐38 and MK‐1 cells at 24 h. G and H, Migration distance in each group of YD‐38 and MK‐1 cells. I and J, The number of invasive cells in each group of YD‐38 and MK‐1 cells. ^*^ *P* < .05, ^**^ *P* < .01

### 3.5 *UCA1* facilitates tumor progression in vivo

To further determine the role of *UCA1* in OSCC tumorigenesis in vivo, transfected cells were injected into the nude mice, and we found that *UCA1* silencing significantly suppressed tumor weight and size in xenograft mice; however, overexpressing *UCA1* noticeably accelerated tumor growth, and the effect of *UCA1* was attenuated by miR‐143‐3p (*P* < .01, Figure 7A‐D). Additionally, the protein and mRNA expressions of *MYO6* were significantly reduced in the si‐UCA1 group but elevated in the pc‐UCA1 group, and miR‐143‐3p overturned these functions of *UCA1* (*P* < .01, Figure 7E‐J). Moreover, immunohistochemical staining for *MYO6* was also consistent with the protein and mRNA expressions of *MYO6* (*P* < .01, Figure 8A‐D).

**Figure 7:** LncRNA *UCA1* promotes tumor growth in a xenograft mouse model of OSCC. A‐D, Xenograft tumor was photographed and tumor weight was measured in each group of YD‐38 and MK‐1 cells. E, Western blot analysis of *MYO6* in each group of YD‐38 cells. F, The protein expression of the *MYO6* in YD‐38 cells. G, The mRNA expression of *MYO6* in each group of YD‐38 cells. H, Western blot analysis of *MYO6* in each group of MK‐1 cells. I, The protein expression of the *MYO6* in MK‐1 cells. J, The mRNA expression of *MYO6* in each group of MK‐1 cells. ^*^ *P* < .05, ^**^ *P* < .01

**Figure 8:** LncRNA *UCA1* upregulates *MYO6* in a xenograft mouse model of OSCC. A, Representative immunohistochemical images for *MYO6* of tumor sections from xenograft mice injected with YD‐38 cells (scale bar = 100 μm). B, The staining intensity of *MYO6* by immunohistochemistry. C, Representative immunohistochemical images for *MYO6* of tumor sections from xenograft mice injected with MK‐1 cells (scale bar = 100 μm). D, The staining intensity of *MYO6* by immunohistochemistry. ^*^ *P* < .05, ^**^ *P* < .01

To understand the effect of *UCA1* on the OSCC metastasis, we measured the epithelial‐mesenchymal transition (EMT) markers and two matrix metalloproteinases (MMPs) of the tumor tissues in the mice. When *UCA1* was suppressed, the expression of E‐cadherin (epithelial marker) was notably increased in the mRNA and protein levels, while the N‐cadherin (mesenchymal marker), MMP‐2, and MMP‐9 were downregulated (*P* < .01, Figure 9A‐C). However, when *UCA1* was upregulated, the expression patterns of these molecules were the opposite (*P* < .01, Figure 9D‐F).

**Figure 9:** LncRNA *UCA1* promotes EMT makers in a xenograft mouse model of OSCC. A, Western blot of EMT makers in each group of tumors from xenograft mice injected with YD‐38 cells. B and C, The protein and mRNA levels of the EMT makers in tumors from xenograft mice injected with YD‐38 cells. D, Western blot of EMT makers in each group of tumors from xenograft mice injected with MK‐1 cells. E and F, The protein and mRNA expression of the EMT makers in tumors from xenograft mice injected with MK‐1 cells. ^*^ *P* < .05, ^**^ *P* < .01

## 4 DISCUSSION

Evidence indicated that lncRNAs are vital regulators in physiological process of cancers.^24^, ^25^ However, there are still limited studies performed on lncRNAs in OSCC. Therefore, it is urgent to determine the molecular mechanism of OSCC progression and discover effective therapy targets based on lncRNA.

Dysregulation of lncRNAs, including *HOXA11‐AS*, *LEF1‐AS1*, and *TUG1*, is involved in OSCC progression.^26^, ^27^, ^28^ Moreover, lncRNA *ADAMTS9‐AS2* can promote tongue squamous cell carcinoma proliferation, migration, and EMT.^29^ However, the roles of lncRNAs in OSCC progression have not been clearly elucidated. Herein, we investigated the potential effect of the lncRNA *UCA1* on OSCC, and found that *UCA1* promotes OSCC cell proliferation, migration, and invasion in vitro and in vivo, suggesting that it could be a potential therapeutic target for treating OSCC.

Studies suggest that *UCA1* serves as an oncogene in various human cancers, for instance, it promotes the growth of adrenocortical cancer cells, while silencing *UCA1* can inhibit hemangioma cell growth, migration, and invasion.^30^, ^31^ *UCA1* also plays an oncogenic role in nasopharyngeal carcinoma,^32^ osteosarcoma,^33^ colon,^34^ and pancreatic cancer.^35^ Additionally, *UCA1* can act as a potential molecular marker for metastasis and prognosis in multiple cancers.^36^ In our study, *UCA1* increased both in OSCC tissues and cells and promoted OSCC progression in vitro and in vivo.

Moreover, high expression of *UCA1* was associated with lymphatic metastasis and recurrence of OSCC patients. Previous studies showed that EMT plays a pivotal role in tissue metastasis.^37^ LncRNAs are involved in EMT, for instance, the knockdown of lncRNA *SNHG7* suppresses EMT in prostate cancer,^38^ and downregulated *HAGLR* inhibits EMT and metastatic potential in esophageal cancer.^39^ As a result, *UCA1* may be conducive to OSCC metastasis via facilitating the EMT process. To further confirm our speculation, we detected the EMT markers (E‐cadherin and N‐cadherin) and MMPs in tumors from xenograft mice, and discovered that E‐cadherin was notably increased but N‐cadherin, MMP‐2, and MMP‐9 were greatly suppressed by si‐UCA1, indicating that the overexpression of *UCA1* can enhance proliferation and EMT to cause an aggressive clinical outcome to OSCC patients.

LncRNAs can act as molecular sponges to miRNAs.^40^ *UCA1* is reported to regulate cancer progression by acting as a sponge for miR‐582‐5p,^41^ miR‐204,^42^ miR‐495‐3p,^43^ and other miRNAs. Therefore, we identified some potential target miRNAs of *UCA1* in OSCC using bioinformatics tools, and miR‐143‐3p was confirmed as a potential target for *UCA1*. Previous reports have revealed that miR‐143‐3p inhibits colorectal cancer metastases by targeting *ITGA6* and *ASAP3*.^44^ In addition, miR‐143‐3p suppresses the growth and invasiveness of melanoma cells by targeting cyclooxygenase‐2.^45^ Furthermore, miR‐143‐3p can be targeted by other lncRNAs, including *ADAMTS9‐AS2*,^46^ *OIP5‐AS1*,^47^ and *OECC*,^48^ to inhibit tumor cell invasion and migration. Herein, we found that miR‐143‐3p mimics exerted an inhibitory effect on the OSCC cell growth and metastasis and was related to lymphatic metastasis and recurrence of patients with OSCC.

We discovered that miR‐143‐3p suppressed OSCC progression via targeting *MYO6*. The data revealed that *MYO6* exhibited a tumor‐promoting property in various cancers, including prostate,^19^ gastric,^21^ breast,^49^ and lung cancer.^50^ Moreover, consistent with previous studies, we observed that *MYO6* is a downstream target for miR‐143‐3p,^51^ and that *MYO6* can also be regulated by lncRNA such as *SOX21‐AS1*.^52^ We also found that *MYO6* was elevated in OSCC tissues and cells, and increased *MYO6* reversed the inhibitory effects of miR‐143‐3p on OSCC cells, suggesting that miR‐143‐3p attenuated OSCC cell proliferation, migration, and invasion by suppressing *MYO6*. However, this study is still incomplete, and we still need to further verify the effect of *MYO6* on EMT of OSCC cells.

## 5 CONCLUSION

In conclusion, our study indicates that *UCA1* expression was significantly elevated in OSCC tissues and cells and was correlated with the metastasis and recurrence of OSCC patients. Moreover, the overexpression of *UCA1* markedly promoted OSCC progression in vitro and in vivo by upregulating *MYO6* expression as a sponge of miR‐143‐3p.

## CONFLICT OF INTEREST

The authors declare no conflict of interest.

## Data Availability

The analyzed datasets generated during the study are available from the corresponding author on reasonable request.
